# Study on Behavior and Bearing Capacity Computation Method of Shallow Rock-Socketed Short Piles Based on the Self-Balanced Loading Test

**DOI:** 10.1155/2022/7272219

**Published:** 2022-03-14

**Authors:** Junxiu Liu, Xianfeng Shao, Xuhui Huang, Guangyong Cao

**Affiliations:** ^1^Anhui Province Key Laboratory of Building Structure and Underground Engineering, Anhui Jianzhu University, Hefei, Anhui 230601, China; ^2^College of Civil Engineering, Anhui Jianzhu University, Hefei, Anhui 230601, China; ^3^State Grid Anhui Electric Power Co., Ltd. Construction Company, Hefei, Anhui 230001, China

## Abstract

The self-balanced loading test is a state-of-art pile testing method, but its suitability to pile bearing capacity determination in transformer substation engineering in mountainous and hilly areas is not yet clear. In this study, a two-dimensional axisymmetric numerical model is established by the PLAXIS software to simulate the behavior and bearing mechanism of shallow rock-socketed short piles based on the self-balanced loading test. The model is first validated by simulating the field tests of two adjacent piles under self-balanced loading. Then the influence factors of the load-displacement curves of piles are analyzed. Thereafter, the mechanical mechanism of the self-balanced loading tests is simulated and compared with the conventional static loading tests. It is observed that the rock modulus, rock-socketed depth of piles, and burial depth of the Osterberg Cell affect the load-displacement significantly, but the cohesion of the rocks affects little. Moreover, compared with the conventional static loading tests, the shear stress of the pile-soil interface distributes less uniformly under self-balanced loading conditions. On this basis, a bearing capacity computation method of shallow rock-socketed short piles based on the self-balanced loading test is proposed.

## 1. Introduction

With the rapid and continuous urbanization, there are more and more transformer substation engineering, as important urban infrastructures, constructed in mountainous and hilly areas. Rock-socketed piles with small diameter (generally 600–800 mm), short length (generally 10–20 m), and shallow rock-socketed depth (generally 0.5–1.0 times the pile diameter) are usually adopted for transformer substations in these areas in China. The bearing capacity of these piles is usually obtained by the static loading test [1–8]. This method is to apply physical loads to the pile top at specific time intervals and monitor the displacement at the loading point until failure [9]. The static loading test is the most direct, reliable, and widely used testing method to obtain the bearing capacity of piles, but has some disadvantages such as high cost, heavy workload, and long testing period in particular for high capacity piles [7–10]. For the mountainous and hilly areas with complex geological conditions, it is difficult to transport concrete blocks or sandbags needed for providing adequate reactive capacity for static loading tests. Besides, adverse environmental problems such as vegetation destruction, solid waste generation, energy consumption, and carbon emission may occur in the stacking loading process. Therefore, the application of the conventional static loading test in transformer substation engineering in mountainous and hilly areas is not cost-efficient and environmentally friendly. More economical and sustainable pile testing methods for transformer substation engineering in mountainous and hilly areas are needed.

The self-balanced loading test also referred to as the Osterberg Cell loading test, firstly introduced into engineering practice by Osterberg in Northwestern University [11], is an advanced pile testing approach. When this method is used for pile testing, a particularly designed loading device called Osterberg Cell is placed at the specified position inside piles. The Osterberg Cell is a hydraulic jack-like device with displacement transducer wires extended to the ground surface. During the testing process, the Osterberg Cell is pressurized internally and expanded in a vertical direction [12–16]. Thus, an upward and a downward force inside the pile are generated, and the displacement of the two parts of the pile (above and below the Osterberg Cell) is measured. The actual applied load is in equilibrium with frictions between the upper segment of the pile and the soil, self-weight of the pile, frictions between the lower segment of the pile and the soil, and pile-end resistance. Therefore, dead weight or reaction frame is not required in the self-balanced loading test. The bearing capacity can be obtained from two load-displacement curves of the upper and the lower segment of the pile [17–31].

Compared with the conventional static loading test, the self-balanced method has many advantages. Firstly, because the multilevel Osterberg cell test is frequently employed and over one hydraulic jack can be installed on the same level, the capability of the self-balanced loading test can meet the requirements of almost all piles [22]. Secondly, for the piles with very high design loads, a conventional static loading test needs a very large weighted platform or very strong frame for reaction, which has been prohibitively costly and also difficult to arrange in the available time and space [13]. However, the self-balanced method is economic since a smaller testing area and less testing period and is particularly suitable for areas where a conventional static loading test is difficult to arrange in space. Thirdly, the self-balanced loading test has advantages even in the places where the conventional static loading test can be performed, such as less solid waste and other environmental impacts. Therefore, the self-balanced method is considered a more sustainable pile testing method [32].

Nowadays, the self-balanced loading test has been used for high-rise buildings, bridges, and offshore engineering projects [22–24]. However, there are still many problems not addressed. Firstly, when using the self-balanced loading test, the equilibrium point of the testing pile must be determined before Osterberg Cell placement. But engineering practice shows that it is difficult to estimate the equilibrium points accurately, which fails in the upper and lower segments of the piles to reach the ultimate bearing capacity simultaneously in the self-balanced loading test. Secondly, the loading point and loading mode of the self-balanced method is different from the actual stress condition, resulting in different frictional resistance distribution at the pile-soil interface [16, 17]. In addition, rock-socketed piles used in transformer substation engineering in mountainous and hilly areas usually have lower bearing capacity compared with other engineering projects because of smaller diameter, shorter length, and shallower rock-socketed depth. Therefore, the uplift bearing capacity of the pile will be obviously reduced if the Osterberg Cell is installed inside the pile body. In this study, a two-dimensional axisymmetric numerical model is established by the PLAXIS software to investigate the behavior and bearing mechanism of shallow rock-socketed short piles based on the self-balanced loading test. The model is first validated by simulating the field tests of two adjacent piles under self-balanced loading located in southern Anhui, China. Then the influence factors of the load-displacement curves of piles are analyzed. Thereafter, the mechanical mechanism of the self-balanced loading tests is simulated and compared with the conventional static loading tests. On this basis, a bearing capacity computation method of shallow rock-socketed short piles based on the self-balanced loading test is proposed. The simulation results and computation method should provide valuable information for managers to improve the efficiency of management of transformer substation engineering in mountainous and hilly areas.

## 2. Numerical Modeling

### 2.1. Description of the Field Test

The field tests were carried out to investigate the behavior of two adjacent cast-in-place concrete piles under self-balanced loading in a 500 kv transformer substation engineering located in southern Anhui, China. The length and diameter of the piles were 16.8 m and 0.6 m, respectively. The rock-socketed depth of the piles was 0.7 m.

The subsoil profile of the construction site consists of 4 soil layers. The 4 soil layers from top to bottom are as follows: compacted fill (10.8 m thick), clay (4.6 m thick), gravel (0.7 m thick), and limestone (3.6 m thick). There is no groundwater on the site. The material properties are illustrated in Table 1.

Figure 1 shows the details of the testing pile, ground condition, the Osterberg Cell, and the displacement monitoring system. The Osterberg Cell was located at the pile end and loaded through the loading system above ground. The displacement bars were connected to the upper or lower loading plates of the Osterberg Cell. Multi-stage loading was adopted for the pile testing. The first loading of the test was set to 260 kN, and the loading increment for each stage was set to 130 kN. During the test, each level of loading was maintained until the pile deformation was stable. For the Osterberg Cell selected for the field test, the maximum loading capacity was 2500 kN and the maximum loading stroke was 100 mm.

Figure 2 shows the measured upward displacement of pile bodies (UDPB) and downward displacement of pile ends (DDPE) of the two adjacent piles (A1 and A2) during the self-balanced loading test. It can be seen that their load-displacement curves were generally coincident, indicating that the self-balanced loading tests have good repeatability. During the field tests, when loaded to the 15th grade (2080 kN), the UDPB and DDPE of A1 were 4.10 mm and 77.06 mm; and the UDPB and DDPE of A2 were 4.81 mm and 71.88 mm. The total displacement nearly reached the maximum loading stroke of the Osterberg Cell and therefore the loading was stopped.

### 2.2. Finite Element Mesh and Boundary Conditions

The finite element software PLAXIS is adopted in this study. PLAXIS is developed by the Delft University of Technology and could be used to simulate the nonlinear, time-dependent, and anisotropic behavior of soils and rocks [33].  Figure 3 shows the two-dimensional axisymmetric numerical model of the self-balanced loading test. The axis of symmetry is set at the axis of the pile. The boundary conditions are taken as rollers on the vertical boundary surfaces of the model and as fully fixed at the base of the model [34]. In the numerical model, the upper and lower loading plates of the Osterberg Cell are represented by two uniform distributed loads. In other words, the stress and displacement of the pile are simulated by applying upward and downward uniformly distributed loads to the upper and lower segments of the pile, respectively. The finite element mesh is set to be fine and automatically divided by the PLAXIS software. As shown in Figure 3, the interface elements of PLAXIS are used to simulate the interaction between the pile body and soils.

### 2.3. Material Parameters

The hardening-soil (HS) model is adopted for the soils and rock. The HS model is an advanced Duncan–Chang model. The yield surface of the HS model is not fixed but can expand with plastic straining, and the hardening modes consist of compression hardening and shear hardening [33, 35].

In the HS model, the confining stress dependent stiffness modulus *E*_50_, which is corresponding to the 50% ultimate deviatoric stress, is used to account for the hyperbolic stress-strain relation in primary loading and is given by the equation:

(1) $$\begin{array}{c} E_{50}=E_{50}^{ref}{\left(\frac{c\;\cos\;\varphi -\sigma_{3}^{\prime }\sin\;\varphi }{c\;\cos\;\varphi +p^{ref}\sin\;\varphi }\right)}^{m}, \end{array}$$

where *p*^*ref*^ is a reference pressure and the default setting of *p*^*ref*^ in PLAXIS is 100 kPa; *E*_50_^*ref*^ is a reference stiffness modulus under the reference confining pressure of *p*^*ref*^; *σ*_3_′ is the confining pressure in a triaxial test; *m* is the power for the stress-level dependency of stiffness.

The unloading/reloading stiffness (*E_ur_*) can be expressed as

(2) $$\begin{array}{c} E_{ur}=E_{ur}^{ref}{\left(\frac{c\;\cos\;\varphi -\sigma_{3}^{\prime }\sin\;\varphi }{c\;\cos\;\varphi +p^{ref}\sin\;\varphi }\right)}^{m}, \end{array}$$

where *E*_*ur*_^*ref*^ is the reference unloading/reloading stiffness corresponding to the confining stress *p*^*ref*^.

Table 2 summarizes the values of the constitutive parameters of the soils used in the numerical simulation. The constitutive parameters for the HS model are obtained by using the following empirical relationships: *E*_*ur*_^*ref*^=3*E*_*oed*_^*ref*^=3*E*_50_^*ref*^, in which *E*_*oed*_^*ref*^  = tangent stiffness for primary oedometer loading [33]. For simplicity, *m* is assumed to be 0.5.

### 2.4. Modeling Procedure

The modeling procedures were the same as the field tests: (1) Define the material properties of the numerical model; (2) Initiate the boundary and initial stress conditions, and the initial equilibrium state; (3) Activate the pile and the interface elements between the pile body and soils, and calculate to the equilibrium state; (4) Activate the upward and downward uniformly distributed loads to the upper and lower segments of the pile. The uniformly distributed load started at 260 kN and gradually increased to 2080 kN in 15 grades, that is, the corresponding stress on the loading surfaces increased from 920 kPa to 7360 kPa. Each grade of the loading was calculated until mechanical equilibrium and displacement stability.

### 2.5. Numerical Results

#### 2.5.1. Deformation

Figure 4 shows the computed displacement contour and deformed mesh of the numerical model under the self-balanced loading of 2080 kN, in which the deformed mesh is magnified by 10 times. According to Figure 4(a), the largest displacement occurs at the pile end (over 100 mm) while the upward displacement of the pile body is very small (less than 10 mm). As shown in Figure 4(b), although there is relative sliding between the pile body and the surrounding soil along with the pile-soil interface, the sliding momentum is small. The rock at the pile end deforms greatly than the pile body, indicating that the end bearing resistance of the pile is more fully developed than the side friction resistance.

#### 2.5.2. Load-Displacement Curves

Figure 5 compares the displacement curves obtained from the field testing measurements and numerical simulations. It can be found that the DDPE (80 mm) is obviously larger than UDPB (10 mm) and the two groups of load-displacement curves are both approximately linear. The simulation results are in good agreement with the field testing measurements, indicating that the developed numerical model is reasonable and can be used to simulate the self-balanced loading test.

## 3. Sensitivity Analysis

The influences of different rock modulus, rock cohesion, rock-socketed depth of pile, and Osterberg Cell burial depth on the load-displacement curves of piles under self-balanced loading were analyzed. To simplify the analysis process, the foundation soil was assumed to contain two layers of soil: the upper layer was the 20 m thick soil and the lower layer was the 20 m thick rock. The length of the pile was 21 m, of which the rock-socketed depth was 1.0 m. The Osterberg Cell was located at the pile end initially. The parameters of the soil and rock are simplified and shown in Table 3.

### 3.1. Rock Modulus

Figure 6 compares the load-displacement curves of the self-balanced loading test piles under different rock modulus. The representative modulus *E* is set to be 40, 80, 120, and 240 MPa, respectively. The secant and tangent stiffness (*E*_50_^*ref*^ and *E*_*oed*_^*ref*^) of the HS model is assumed to be equal to the representative modulus *E*, and the unloading/reloading stiffness *E*_*ur*_^*ref*^ is three times the representative modulus (i.e., 120, 240, 360, and 720 MPa). It can be found that when the rock modulus increases from 40 MPa to 240 MPa, the DDPE decreases from 96 mm to 16 mm, while the curves of the UDPB approximately coincides. This means that the deformation modulus of rocks has significant impacts on the DDPE but little impact on the UDPB under the self-balanced loading.

### 3.2. Rock Cohesion

Figure 7 compares the load-displacement curves of the self-balanced loading test piles under different rock cohesion. The value of the cohesion *c* is set to 20, 40, and 80 kPa, respectively. It can be seen that the load-displacement curves under different rock cohesion approximately coincide, indicating that only compression deformation is developed in the rocks but shear failure does not occur.

### 3.3. Rock-Socketed Depth of the Pile

Figure 8 compares the load-displacement curves of the self-balanced loading test piles under different rock-socketed depths. The rock-socketed depth is set to be 1.7*D*, 3.3*D*, 5.0*D*, and 6.7*D* (*D* is the diameter of the pile, and *D* = 0.6 m), respectively. It can be seen that the rock-socketed depth has a significant influence on the load-displacement curves of the self-balanced loading test piles. When the load is small, the load-displacement curves of different rock-socketed depths basically coincide. As the rock-socketed depth increases, the side resistance of the pile body and the end bearing capacity of the pile end increase correspondingly.

### 3.4. Osterberg Cell Burial Depth

Figure 9 compares the load-displacement curves of the self-balanced loading test piles under different burial depths of the Osterberg Cell. The burial depth of the Osterberg Cell (*H*) is set to be 20, 18, 16, and 14 m, respectively. It can be seen that the burial depth of the Osterberg Cell affects the load-displacement curves obviously. When the Osterberg Cell is located at the pile end, the UDPB is small and the downward displacement of the lower plate of the Osterberg Cell (DDLP) increases approximately linearly with the load. Both the side friction resistance of the upper segment of the pile and the end bearing resistance of the pile end have not reached the ultimate state. When the burial depth of the Osterberg Cell decreases, the DDLP is also decreased. The UDPB varies not obviously when the load is small with the burial depth of the Osterberg Cell decreasing. However, there exists a critical load. When exceeding the critical load, the upward displacement of the pile body increases significantly, indicating that the side friction resistance has reached the ultimate state. The shallower the Osterberg Cell set, the lower the critical load is.

## 4. Comparison with the Conventional Static Loading Test

The load-displacement curves and stress states of self-balanced loading test piles are different from the conventional static loading test piles. Comparative studies were carried out based on the validated numerical model to investigate the displacement and mechanical performance of the piles under self-balanced loading, static uplift loading, and static compressive loading. The geometric size of the numerical model was the same as those in Section 3, and the Osterberg Cell was located at the pile end. The static uplift loading and compressive loading were applied on the top of the pile. The constitutive parameters of the numerical model were shown in Table 3.

### 4.1. Self-Balanced Loading and Static Uplift Loading

Figure 10 compares the upward displacement of piles under self-balanced loading and static uplift loading. It can be found that both curves are approximately linear when the load is not large. But when the load exceeds a critical value, the displacements of the piles suddenly increase. These critical loads, which are basically equal under the two loading conditions, can be regarded as the ultimate uplift bearing capacity of the piles. Therefore, the self-balanced loading test can precisely determine the uplift bearing capacity of shallow rock-socketed short piles.

In addition, the upward displacement of the pile under the self-balanced loading is slightly larger than that of the pile under the static uplift loading. Therefore, when the self-balanced loading tests are used to determine the displacement of piles under uplift loading, the results are biased towards safety.

Figure 11 compares the shear stress distribution of the pile-soil interface of the piles under the self-balanced loading and static uplift loading. The interface shear stresses under the two loading conditions are both downward. As shown in Figure 11, when the load is small, the distributions of the shear stress under the two loading conditions are basically coincident. Increasing the applied load will increase the interface shear stress. The minimum shear stress is located at the pile top and the maximum shear stress is at the pile end. This is because the shear stress of the pile-soil interface is related to the shear strength of the surrounding soil. The greater the depth, the greater the horizontal earth pressure, which increases the shear strength of the interface.

It can be also found that the shear stress of the pile-soil interface is distributed more uniformly under the static uplift loading when the load is less than 2080 kN. Specifically, the interface shear stress of the upper half part under the static uplift loading is larger than that under the self-balanced loading, and the lower half part is the opposite. This is because the shear stress of the pile-soil interface is also related to the relative displacement between the pile and soils. The static uplift loading is applied to the pile top, and the relative displacement between the pile and soils is the largest at the pile top and decreased with depth. However, the self-balanced loading is applied to the pile end and the relative displacement is also the largest at the pile end. Therefore, the interface shear stress of the lower half part under the self-balanced loading is larger than that under the static uplift loading.

When the load reaches 2080 kN, the interface shear stresses under the two loading conditions become a consistent distribution, indicating that the shear strength of the pile-soil interface is fully developed and the testing piles all reach the ultimate state. However, the curve of interface shear stress under static uplift loading is not smooth because a larger slip occurs between the pile and soil.

### 4.2. Self-Balanced Loading and Static Compressive Loading

Figure 12 compares the load-displacement curves of the piles under the self-balanced loading and static compressive loading. It can be seen that the displacement of the static compressive loading pile is significantly smaller than the DDPE of the self-balanced loading test pile. The UDPB of the self-balanced loading test pile keeps linear when the load is not large. But there exists an ultimate load, beyond which the displacement increases obviously.

Figure 13 compares the shear stress distribution of the pile-soil interface of the piles under the self-balanced loading and static compressive loading. The direction of the interface shear stress under the self-balanced loading is downward, while the direction of the interface shear stress under the compressive loading is upward.

As shown in Figure 13, when the load is small, the distributions of the interface shear stress under the self-balanced loading and compressive loading are basically coincident. Increasing the applied loads will increase the interface shear stress. The minimum shear stress is located at the pile top and the maximum is located at the pile end. The shear stress of the pile-soil interface is distributed more uniformly under static compressive loading conditions. These are also because the shear stress distribution of the pile-soil interface is related to the shear strength of the surrounding soil and the relative displacement between the pile and soil.

However, when the load is increased from 2820 kN to 3100 kN, the interface shear stress of the piles under the compressive loading changes not significantly. This is due to the effect of the pile-end resistance.

## 5. A Bearing Capacity Computation Method of Piles

Based on the statistics of the numerical simulation results, a bearing capacity computation method of the shallow rock-socketed short piles under the self-balanced loading is established. In this method, the Osterberg Cell is set at the pile end and the ultimate compressive bearing capacity of the pile can be calculated by

(3) $$\begin{array}{c} Q_{u}=Q_{uu}+Q_{ud}, \end{array}$$

where *Q*_*u*_ represents the compressive bearing capacity of the pile; *Q*_*uu*_ represents the ultimate side resistance of the pile (the load corresponding to the inflection point of the load-displacement curve of UDPB); and *Q*_*ud*_ represents the pile end bearing capacity corresponding to the allowable settlement of 40 mm.

Figure 14 shows the load-displacement curves computed by the numerical modelings under the compressive and self-balanced loading conditions. The pile length varies from 14 m to 20m. As shown in Figure 14(a), the static compressive test-based ultimate bearing capacities corresponding to the allowable settlement of 40 mm are 2990, 3370, 4050, and 4300 kN for the different pile lengths of 14, 16,18, and 20 m. According to Figure 14(b), for different pile lengths of 14, 16, 18, and 20 m, the ultimate side resistances *Q*_*uu*_ are 1710, 2130, 2610, and 3000 kN, and the pile end bearing capacities *Q*_*ud*_ are 1090, 1110, 1150, and 1200 kN. The ultimate compressive bearing capacities of the piles determined by the proposed computation method are 2800, 3240, 3760, and 4200 kN.

Figure 15 shows the ultimate bearing capacity obtained from the numerical simulation results under the two loading conditions. The results based on the field test measurements are also shown in Figure 15. It can be seen that the ultimate bearing capacities of these two methods are approximately consistent. Therefore, the proposed bearing capacity computation method of the shallow rock-socketed short piles under the self-balanced loading is reliable.

## 6. Conclusions and Recommendations

In this study, a two-dimensional axisymmetric numerical model is established by the PLAXIS software to investigate the behavior and bearing mechanism of shallow rock-socketed short piles based on the self-balanced loading test. The model is first validated by simulating the field tests of two adjacent piles under self-balanced loading located in southern Anhui, China. Then the influence factors of the load-displacement curves of piles are analyzed. Thereafter, the mechanical mechanism of the self-balanced loading tests is simulated and compared with the conventional static loading tests. On this basis, a bearing capacity computation method of shallow rock-socketed short piles based on the self-balanced loading test is proposed. The simulation results and computation method should provide valuable information for managers to improve the efficiency of management of transformer substation engineering in mountainous and hilly areas. The following conclusions can be drawn:

1. The side resistance and end bearing of the pile increase with the rock-socketed depth. Downward displacement of pile end will decrease with the decrease of the burial depth of the Osterberg Cell. Increasing the rock modulus will also decrease the downward displacement of the pile end but has little impact on the upward displacement of the pile body. However, the rock cohesion has little effect on the load-displacement curve of the piles.
2. Compared with self-balanced loading test piles, the shear stress of the pile-soil interface distributes more uniformly under static uplift or compressive loading conditions. The interface shear stress of the upper half part of the pile under the self-balanced loading test is larger than that under static uplift or compressive loading, and the lower half part is the opposite.
3. For the self-balanced loading test of the shallow rock-socketed short piles, the Osterberg Cell is recommended to be set at the pile end. The ultimate uplift bearing capacity of the piles can be directly determined by the inflection point of the load-displacement curve of the pile body. The ultimate compressive bearing capacity of the piles is the sum of the ultimate side resistance and the end bearing capacity corresponding to the allowable settlement of 40 mm.

## Figures and Tables

**Figure 1:** Details of the field test. (a) Pile and ground condition. (b) The Osterberg Cell and displacement monitoring.

**Figure 2:** Measured load-displacement curves of the two adjacent piles.

**Figure 3:** Axisymmetric numerical model of the self-balanced loading test.

**Figure 4:** Simulated deformation of the testing pile and surrounding soils under self-balanced loading. (a) Displacement contour. (b) Deformed mesh.

**Figure 5:** Load-displacement curves of the field testing measurements and numerical simulations.

**Figure 6:** Load-displacement curves under different rock modulus.

**Figure 7:** Load-displacement curves under different rock cohesion.

**Figure 8:** Load-displacement curves under different rock-socketed depths of the pile.

**Figure 9:** Load-displacement curves under different burial depths of the Osterberg Cell.

**Figure 10:** Load-displacement curves of piles under the self-balanced loading and uplift loading.

**Figure 11:** Shear stress distributions of the pile-soil interface under the self-balanced loading and uplift loading.

**Figure 12:** Load-displacement curves of piles under the self-balanced loading and compressive loading.

**Figure 13:** Shear stress distributions of the pile-soil interface under the self-balanced loading and compressive loading.

**Figure 14:** Load-displacement curves for different loading conditions. (a) Compressive loading. (b) Self-balanced loading.

**Figure 15:** Comparison of the pile bearing capacity from the self-balanced and compressive loading tests.

**Table 1:** Summary of the subsoil properties.

Material	Layer 1	Layer 2	Layer 3	Layer 4
*γ* (kN·m^−3^)	17.8	19.5	19.8	22.0
*ω* (%)	18.0	24.0	19.0	–
*e*_0_	0.80	0.55	0.60	–
*E*_50_^*ref*^ (MPa)	22.0	18.0	23.0	43.5
*c* (kPa)	16.0	20.0	25.0	23.0
*φ* (°)	30.0	27.0	30.0	42.0

Note: *γ* = unit weight; *ω* = water content; *e*_0_ = initial void ratio; *E*_50_^*ref*^  = secant modulus in standard drained triaxial testing; *c* = cohesion; *φ* = friction angle.

**Table 2:** Model parameters of the subsoil.

Material	Layer 1	Layer 2	Layer 3	Layer 4
Material model	HS	HS	HS	HS
*γ* (kN·m^−3^)	17.8	19.5	19.8	22.0
*E*_50_^*ref*^ (MPa)	22.0	18.0	23.0	43.5
*E*_*oe* *d*_^*ref*^ (MPa)	22.0	18.0	23.0	43.5
*E*_*ur*_^*ref*^ (MPa)	66.0	54.0	69.0	130.5
*m*	0.5	0.5	0.5	0.5
*ν*_ur_	0.2	0.2	0.2	0.2
*c* (kPa)	16.0	20.0	25.0	23.0
*φ* (°)	30.0	27.0	30.0	42.0

Note: *E*_*oed*_^*ref*^  = tangent stiffness for primary oedometer loading; *E*_*ur*_^*ref*^  = unloading/reloading stiffness; *m* = power for stress-level dependency of stiffness; *ν*_ur_ = Poisson's ratio for unloading-reloading.

**Table 3:** Simplified model parameters.

Material	*γ* (kN·m^−3^)	*E*_50_^*ref*^ (MPa)	*E*_*oed*_^*ref*^ (MPa)	*E*_*ur*_^*ref*^ (MPa)	*c* (kPa)	*φ* (°)
Soil	17.8	22.0	22.0	66.0	16	30
Rock	22.0	40.0	40.0	120.0	23	42

## Data Availability

The data that support the findings of this study are available from the corresponding author upon reasonable request.
